# Open reduction and closed reduction internal fixation in treatment of femoral neck fractures: a meta-analysis

**DOI:** 10.1186/1471-2474-15-167

**Published:** 2014-05-22

**Authors:** Weiguo Wang, Junjie Wei, Zhanwang Xu, Wenkun Zhuo, Yuan Zhang, Hui Rong, Xuecheng Cao, Pingshan Wang

**Affiliations:** 1 Department of Orthopaedic Surgery, General Hospital of Jinan Military Command, 250031 Jinan, China; 2 Research on 2013 stage doctoral student of TCM Orthopaedics, Shandong University of Traditional Chinese Medicine, Jinan, China; 3 Outpatient Department, General Hospital of Jinan Military Command, 250031 Jinan, China; 4 Department of Orthopaedics, The First Affiliated Hospital of Shandong University of Traditional Chinese Medicine, NO.16369, Jingshi Road, 250014 Jinan, China

**Keywords:** Femoral neck fracture, Open reduction internal fixation, Closed reduction internal fixation

## Abstract

**Background:**

A meta-analysis was performed to assess the association between healing rate, avascular necrosis (AVN) of femoral head and two reductions-open reduction internal fixation (ORIF) and closed reduction internal fixation (CRIF) for femoral neck fracture.

**Methods:**

A literature-based search was conducted to identify all relevant studies published before September 10, 2013. The odd ratio (OR) and 95% confidence interval (CI) were used for estimating the effects of the two reduction methods. Data were independently extracted by two investigators who reached a consensus on all of the items. The heterogeneity between studies was examined by χ^2^-based Q statistic. Egger’s regression analysis was used to evaluate publication bias. Statistical analysis was performed by Stata 10.0 software.

**Results:**

We examined 14 publications. The results of the present meta-analysis showed that AVN of femoral head were significant associated with the two reductions (CRIF vs. ORIF, OR = 1.746, 95% CI 1.159-2.628, p = 0.008), while the healing rate were not (CRIF vs. ORIF, OR = 0.853, 95% CI 0.573-1.270, p = 0.433).

**Conclusion:**

The present meta-analysis indicated the risk of AVN of femoral head was significant higher after CRIF fixation compared with ORIF, but no association between the healing rate and the two reductions for femoral neck fracture.

## Background

Femoral neck fracture, known as hip fracture, occurs in the proximal end of the femur near the hip, and is often due to osteoporosis [1]. The incidence of femoral neck fracture is increasing at an exponential rate as a result of the longevity of the general population [2]. It is one of the most common consequences of injuries in the elderly population [3]. Despite advances in surgical techniques and medical care, the risk of nonunion and avascular necrosis (AVN) of femoral head after fixation have not changed appreciably in the last 50 years [4].

Emergency internal fixation is one of the main options for the treatment of displaced femoral neck fractures [5]. It contains open reduction internal fixation (ORIF) and closed reduction internal fixation (CRIF). Both of the two methods have their advantages and disadvantages [6]. Although ORIF has advantages of direct look and restoration of normal function, its application still limited by the potential negative effects of nerve damage, swelling, incomplete healing of the bone, increased pressure and blood clot [7]. CRIF has advantages of avoiding injury to the medial circumflex femoral artery [8]. However, intracapsular pressure formed by CRIF compromised femoral head circulation, and prolonged extension and internal rotation position on the fracture table reduced the blood supply to the femoral head, what’s more, the repeated forceful manipulation increased the risk of AVN [6]. Thus, the optimal treatment of femoral neck fractures remains controversial [9]. The purpose of the present meta-analysis was to compare the healing rate and incidence of AVN postoperative between ORIF and CRIF.

## Methods

### Search strategy

PubMed, MEDLINE, PMC, Embase, Vipbrowser database (http://www.cqvip.com/) and Wanfang database (http://www.wanfangdata.com.cn/) on line were searched using “open reduction”, “closed reduction” and “femoral neck fracture” as key words. There was no language restriction. The search was completed on September 10, 2013.

### Inclusion and exclusion criteria

All of the studies identified were reviewed by two investigators independently, any dispute being resolved by discussion. The inclusion and exclusion criteria were as follows: First, each study was randomized controlled trial and had been published as an original study. Second, if the data were duplicated and had been published more than once, the most recent and complete study was chosen. Third, the following were excluded: review articles, abstracts, editorials, reports with incomplete data.

### Data extraction

Data were independently extracted by two investigators who reached a consensus on all of the items. Information extracted from each study was considered as follows: name of first author, publication year, ethnic origin of the population studied, number of participants in case and control groups.

### Statistical analysis

The heterogeneity between studies was examined by χ^2^-based Q statistic [10] and I^2^ test. The p value of Q statistic less than 0.05 and/or I^2^ more than 50% was considered significantly heterogeneous, otherwise there was no significant heterogeneity. Pooled odd ratios (ORs) and 95% confidence intervals (CIs) were computed by the fixed-effects method of Mantel-Haenszel (Peto method) under no heterogeneity between studies. If significant heterogeneity existed between studies, then a random effects model of DerSimonian-Laird (D-L method) was applied for data synthesis. Egger's regression analysis was used to evaluate the publication bias. A p value less than 0.05 was considered statistically significant. Statistical analysis was performed by Stata 10.0 software.

## Results

### Data selection

The data selection process was displayed in Figure 1. By the computer search of the electronic databases, totally 820 papers were observed. A total of 126 duplicates and 27 reviews were excluded. By reviewing of the title and abstract, 567 articles were rejected for obvious unmatched with the inclusion and exclusion criteria. Then the full texts of 27 potential citations were downloaded for further selection and 13 citations were excluded by incomplete data. Finally, 14 studies [11-24] were included in this study.

**Figure 1:** The process of data selection.

### The healing rate of ORIF and CRIF

A total of nine studies [11-19] met the inclusion and exclusion criteria in the meta-analysis of healing rate of ORIF and CRIF (Table 1), which contained 405 patients of ORIF and 442 patients of CRIF. Egger’s regression analysis indicated no publication bias (p = 0.462). No significant heterogeneity was observed among studies (p = 0.462), so a fixed effect model was used and generated a combined OR of 0.853 (95% CI 0.573-1.270). Meta-analysis showed that no significant association between the healing rate and the two reductions (p = 0.433), and the forest plot was presents at Figure 2.

**Table 1:** Characteristics of studies included in the meta-analysis of the nonunion rate between the two groups

**Study**	**Year**	**ORIF**		**CRIF**	
		**Union**	**Nonunion**	**Union**	**Nonunion**
Liu [11]	2003	21	21	33	23
Wang [12]	2005	19	1	41	1
Song [13]	2010	14	1	7	5
Zhang [14]	2011	47	3	48	2
Ye [15]	2011	16	12	19	13
Lin [16]	2012	18	1	12	3
Zhou [17]	2012	124	13	113	8
Xia [18]	2013	37	3	33	3
Zhang [19]	2013	43	11	68	10

ORIF, open reduction internal fixation; CRIF, closed reduction and internal fixation.

**Figure 2:** **Forest plots of meta-analysis ofnonunion rate.** Closed reduction internal fixation vs. open reduction internal fixation.

### The AVN of ORIF and CRIF

A total of eleven studies [11,12,14,16-18,20-24] met the inclusion and exclusion criteria in the meta-analysis between AVN and the two reductions (Table 2), which contained 478 patients of ORIF and 505 patients of CRIF. Egger regression analysis indicated no publication bias (p = 0.257). No significant heterogeneity was observed among studies (p = 0.507), so a fixed effect model was used and generated a combined OR of 1.746 (95% CI 1.159-2.628). Meta-analysis showed that significant association between AVN and the two reductions (p = 0.008), and the forest plot was presents at Figure 3.

**Table 2:** Characteristics of studies included in the meta-analysis of AVN between the two groups

**Study**	**Year**	**ORIF**		**CRIF**	
		**Normal**	**AVN**	**Normal**	**AVN**
Liu [11]	2003	40	2	53	3
Upadhyay [20]	2004	36	8	41	7
Wang [12]	2005	18	2	41	1
Gao [21]	2008	25	3	37	5
Zhang [14]	2011	49	1	48	2
Kan [22]	2011	44	5	53	20
Kamal [23]	2011	15	3	8	3
Lin [16]	2012	19	0	13	2
Zhou [17]	2012	126	11	104	17
Xia [18]	2013	37	3	27	9
Mohammad [24]	2013	26	5	9	2

ORIF, open reduction internal fixation; CRIF, closed reduction and internal fixation.

**Figure 3:** **Forest plots of meta-analysis of the risk of AVN.** Closed reduction internal fixation vs. open reduction internal fixation.

## Discussion

Femoral neck plays an important in weight bearing and movement. ORIF and CRIF are the two common techniques to cure femoral neck fracture. The results of the present meta-analysis showed that there was significant difference of AVN between ORIF and CRIF, while the healing rate was not.

AVN of femoral head remains a major complication of femoral neck fractures [25]. It is often occurs when the blood supply to bone is disrupted. Bisphosphonate therapy has been shown to preserve the AVN of femoral head in experimental and short-term clinical studies [26]. Increased oxidative stress is considered one of the main causes of steroid-induced AVN of the femoral head [27]. Intensive bone cell apoptosis contributes to AVN of femoral head [28]. Our meta-analysis indicated the incidence of AVN of femoral head in CRIF was significant higher than ORIF (OR = 1.746, 95% CI 1.159-2.628, p = 0.008). This might be caused by the pressure of CRIF that compromised the blood supply to the femoral head [6].

Nonunion is caused by a combination of unfavorable biomechanical and vascular conditions, ignoring general contraindications, and inadequate internal fixation [29]. It also related to age, the quality of bone and the pattern of fracture [20]. It was reported that the risk of nonunion was higher in female than male [30]. The effect of smoking and alcohol drinking may also influence the rate of nonunion [31]. Our meta-analysis showed that there was no significant difference of the healing rate between CRIF and ORIF (OR = 0.853, 95% CI 0.573-1.270, p = 0.433).

The early treatment of femoral neck fracture is critical. CRIF is prior for patients with good blood perfusion of the femoral head while the ORIF should be se1ected for those with poor blood perfusion [12]. It was reported that gentle closed reduction should be tried first, with a maximum of one or two reduction attempts, which could prevent greater displacement with risk of greater damage to the blood supply [32]. Once the CRIF failed, then ORIF should be performed [33]. However, this may increase the risk of AVN as the result of the present study indicated, thus, ORIF is recommended.

There were several limitations in the present meta-analysis that should be noted. First, publication bias, an inherent limitation of all meta-analyses, may still exist because researchers are less likely to publish negative findings, although Egger’s regression analysis did not suggest publication bias in this study. Second, the confounding variables (age, sex, smoking, or alcohol intake) were not adjusted because most of studies didn’t provide respective OR value or sufficient data for calculating OR. Besides, different types of reduction devices may affect the results. Third, we did not perform subgroup analysis for different type of femoral neck fracture because the classifications varied from different studies including Garden [34], Pauwels [35] and Delbet [36] classification. Despite these limitations, the study is still of great importance for evaluating the effects of two reductions for femoral neck fracture treatment, especially considering the main complication - AVN.

## Conclusion

In conclusion, our meta-analysis suggested that the risk of AVN of femoral head was significant higher after CRIF compared with ORIF, while there was no significant difference of the healing rate between the two reductions. ORIF offers advantage over CRIF in terms of AVN for treatment of the femoral neck fractures.

## Consent

Written informed consent was obtained from the patient for the publication of this report and any accompanying images.

## Competing interests

We certify that regarding this paper, no actual or potential conflicts of interests exist; the work is original, has not been accepted for publication nor is concurrently under consideration elsewhere, and will not be published elsewhere without the permission of the Editor and that all the authors have contributed directly to the planning, execution or analysis of the work reported or to the writing of the paper.

## Authors’ contributions

WW and JW participated in the design of this study, and they both performed the statistical analysis. ZX and YZ carried out the study, together with WZ, collected important background information, and drafted the manuscript. HR, XC, and PW conceived of this study, and participated in the design and helped to draft the manuscript. All authors read and approved the final manuscript.

## Authors’ information

Weiguo Wang and Junjie Wei: The first two authors should be regarded as joint First Authors.

## Pre-publication history

The pre-publication history for this paper can be accessed here:

http://www.biomedcentral.com/1471-2474/15/167/prepub
